RETRACTED

# Related Factor Analysis and Nursing Strategies of Diarrhea in Critically Ill Patients with Enteral Nutrition

**DOI:** 10.1155/2022/8423048

**Published:** 2022-09-21

**Authors:** Donglian Liu, Qinghong Liu, Xiansong Wen

**Affiliations:** ^1^Department of Emergency, Ganzhou People's Hospital, Ganzhou341000, Jiangxi, China; ^2^Department of Nursing, Ganzhou People's Hospital, Ganzhou341000, Jiangxi, China

## Abstract

**Objective:**

To explore the related factors of diarrhea in critically ill patients with enteral nutrition (EN) in the intensive care unit (ICU).

**Methods:**

This single-center retrospective study analyzed the occurrence of intolerant diarrhea in ICU patients receiving EN treatment in our hospital. By collecting clinical data, univariate and multivariate logistic regression analysis was used to screen the risk factors for diarrhea.

**Results:**

Among 120 patients included in the study, 68 (48.33%) had diarrhea. Age (OR = 2.599, *P* = 0.027), use of antibiotics (OR = 3.496, *P* = 0.007), ICU hospitalization time (OR = 1.311, *P* = 0.001), and mechanical ventilation time (OR = 1.273, *P* = 0.035) were all independent risk factors for diarrhea in EN.

**Conclusion:**

Older age, frequent use of antibiotics, long ICU stay, and mechanical ventilation time can lead to diarrhea in ICU patients receiving EN treatment. It is necessary to effectively analyze the above independent factors and implement targeted interventions to improve the incidence of diarrhea in patients.

## 1. Introduction

Intensive care unit (ICU) is a specialized department for intensive care and treatment of critically ill patients in hospitals. Studies have shown that the incidence of malnutrition in ICU is 38%–78% [1] and is associated with poor prognosis. Critically ill patients in the intensive care unit (ICU) have high metabolism, high consumption, and stress state. Therefore, the demand for nutrition increases, but such patients often due to chewing, swallowing, consciousness and other factors lead to abnormal eating and need nutritional support treatment. Enteral nutrition (EN) is an important means of nutritional support for ICU patients [2]. Compared with parenteral nutrition (PN), early application of EN can promote the recovery of gastrointestinal mucosal integrity [3] and is also found to be related to the reduction of infection rate, mortality, and hospitalization time [4]. EN is also a treatment recommended by the European Society for European Society for Clinical Nutrition and Metabolism (ESPEN) [5]. EN in a broad sense refers to the way in which nutrients required by patients are provided orally or through tubes (nasogastric tube, nasointestinal tube, and fistula tube) [6]. However, in the ICU, patients who take food orally have certainty in food composition and time frequency. Therefore, EN mentioned in this study is limited to obtaining nutrients through pipelines, excluding oral or semiautonomous eating. Although EN is beneficial for critically ill patients, it often causes complications during treatment, which can aggravate the patient' s condition and even threaten life. Diarrhea is one of the common manifestations of treatment intolerance. Kozeniecki studies have shown that the incidence of diarrhea in critically ill patients during enteral nutrition can reach 66% [7]. Diarrhea in enteral nutrition may lead to loss of nutrients, acid-base imbalance of water electrolyte, perianal skin rupture, and increase hospitalization time and mortality [8]. Therefore, understanding the related factors of diarrhea in enteral nutrition and implementing corresponding measures can effectively improve the prognosis of severe patients.

RETRACTED

Due to the latest medical development, the cure rate and survival rate of ICU patients have improved. People have higher requirements for the prognosis of such patients and the quality of life after discharge. Therefore, reducing the risk of diarrhea in EN treatment to ensure the quality of treatment is critical for ICU patients. At present, the causes of diarrhea after enteral nutrition therapy in ICU patients are not clear. Most of the epidemiological data on diarrhea in critically ill patients in ICU come from countries other than China, which may not reflect the actual situation in China. Regrettably, this issue has rarely attracted the attention of researchers in China. Based on this, we explored the related factors of diarrhea in ICU patients during EN treatment. The research results are of great significance to guide clinicians to take effective intervention measures and reduce the risk of diarrhea.

## 2. Materials and Methods

### 2.1. Design

This single-center, retrospective study collected data of 120 patients who received EN treatment in ICU of our hospital from November 2020 to November 2021. This study was approved by the institutional ethics committee and carried out with the informed consent of patients.

### 2.2. Patients

Patients receive EN in ICU of our hospital. The inclusion criteria are as follows: the patient's age is ≥18 years old, ICU stay is ≥2 days, in line with EN treatment indications, and complete basic clinical data. Exclusion criteria are as follows: at the end stage of malignant tumor, patients had suffered from diseases with diarrhea symptoms such as irritable bowel syndrome and inflammatory bowel disease, acute gastrointestinal bleeding, intestinal polypectomy, radical resection of esophageal cancer, and other gastrointestinal surgery histories.

RETRACTED

### 2.3. Method of EN

All patients in the ICU stay within 24∼48 h, immediately began to nasal feeding tube enteral nutrition support treatment. The daily calorie intake of patients in this study was 30 kcal/kg d. Enteral nutrient solution was continuously input through a thermostatic heater, and the speed and dose were reasonably adjusted according to the patient's intestinal tolerance. Gastric contents were withdrawn at q6h, and gastric contents greater than 150 ml should be suspended and evaluated again after 2 h.

### 2.4. Precautions for EN Feeding

1. EN implementation process: the bed head raised 30°to 45°
2. Before feeding implementation, ensure that the gastrointestinal tube in place and fixed properly
3. q4h feed 20 ml warm water to wash the pipeline to ensure smooth pipeline
4. Daily oral care to prevent oral infection (ordinary patients: 2 times/day; mechanical ventilation patients: 3 times/day)

### 2.5. Collection of Materials

Collect relevant information through the hospital electronic medical record system. It mainly includes gender, age, BMI, EN treatment days, feeding methods, ICU admission diagnosis, mechanical ventilation use, EN preparation type, hypoproteinemia occurrence, antimicrobial use, acute physiology and chronic health evaluation II (APACHE II), ICU hospitalization time, mechanical ventilation time, EN use, and potassium (K), sodium (Na), chlorine (CI), calcium (Ca), and magnesium (Mg) electrolyte levels.

### 2.6. Grouping

Diagnostic criteria: defecation frequency ≥3 times/d; feces volume ≥200 g/d. According to the Bristol stool classification method, feces were paste or water samples. Nurses and doctors are responsible for the mobile phones of the above information. Before that, they received unified training, including disease definition and data entry. Finally, 58 patients with diarrhea were included in the diarrhea group, and 62 patients without diarrhea were included in the nondiarrhea group.

### 2.7. Statistical Analysis

Statistical Package for Social Sciences software for Windows, version 23.0 (SPSS Inc, Chicago, IL, USA) was used to analyze the data. Quantitative data were expressed as mean ± standard deviation, and *t*-test was performed. The enumeration data are described by various cases and percentages, chi-square test, when 1 ≤ theoretical frequency <5 chi-square values need to be corrected, when the theoretical frequency <1 using the exact probability method. Single-factor and multifactor conditional logistic regression models were used to screen the independent factors affecting diarrhea, OR value and 95% confidence interval of risk were calculated, and *P* values <0.05 was considered statistically significant.

RETRACTED

## 3. Results

### 3.1. Baseline Information

Originally, 124 patients met the criteria, but 5 patients were excluded (Figure 1). Finally, 120 patients were included in the study, including 58 cases of diarrhea, 73 males, 67 patients with hypoproteinemia, 79 patients with antimicrobial drugs, 110 patients with nasogastric tube feeding, and 95 patients with mechanical ventilation. The ventilation time was 7.46 ± 1.95 days, 71 patients aged ≥60 years old, 105 patients with EN treatment for 4 days, and the EN usage for 4 days was (1033.49 ± 206.64) ml. 61.67% of the patients entered ICU for EN treatment due to respiratory diseases (Table 1).

### 3.2. Single Factor Analysis of Diarrhea in ICU Patients with EN Treatment

There were statistically significant differences in age, antibiotic use, ICU hospitalization time, and mechanical ventilation time between the diarrhea group and the nondiarrhea group (*P* < 0.05). In addition, the remaining indicators between the two groups are not statistically significant (Table 2). The number of patients aged ≥60 years who developed diarrhea after EN treatment was much larger than that of those who did not (41 vs 30). Similarly, 58% (46/73) of patients who used antibiotics developed diarrhea (Figure 2). The ICU hospitalization time (*r* = −0.367, *P* < 0.001) and mechanical ventilation time (*r* = −0.232, *P* < 0.011) were negatively correlated with the risk of diarrhea (Figure 3).

### 3.3. Multivariate Analysis of Diarrhea in ICU Patients Undergoing EN Treatment

The results of single factor analysis were statistically significant indicators (age, use of antibiotics, ICU hospitalization time, and mechanical ventilation time) as independent variables, to ICU patients with diarrhea after EN treatment as the dependent variable, assignment (Table 3). Multivariate logistic regression analysis showed that age ≥60 years old (OR = 2.599 (1.112–6.074), *P*=0.027), use of antibiotics (OR = 3.496 (1.416–8.632), *P*=0.007), ICU hospitalization time (OR = 1.311 (1.113–1.544), *P*=0.001), and mechanical ventilation time (OR = 1.273 (1.017–1.593), *P*=0.035) were risk factors for diarrhea in ICU patients with EN, and the difference was statistically significant (*P* < 0.05) (Table 4). In addition, we also found that the cutoff values of ICU hospitalization time and mechanical ventilation time in distinguishing EN diarrhea were 9.5 days and 8.5 days, respectively, and their AUCs in distinguishing diarrhea were 0.710 and 0.632, respectively, *P* < 0.05 (Table 5 and Figure 4).

## 4. Discussion

EN intolerance can be manifested as gastrointestinal reactions such as gastric retention, nausea, vomiting, diarrhea, and aspiration. Diarrhea is one of the manifestations of early enteral nutrition intolerance, which will lead to treatment interruption. In severe cases, it will increase the duration of mechanical ventilation, prolong hospitalization time, even increase the mortality of patients, affect the psychology of patients, and greatly increase the workload of nursing [9]. The incidence of EN intolerance was significantly higher in ICU patients (35.6%) than in general patients [10]. Studying the related factors of diarrhea in ICU patients with enteral nutrition is of great significance to the treatment, prevention, and prognosis improvement of patients.

RETRACTED

According to research reports, intensive care unit patients with diarrhea rate as high as 66% [7]. Weiting chen et al. [11] found that the early diarrhea rate of enteral nutrition in ICU patients was 30.8%. In this study, 120 severe patients were treated with enteral nutrition, and 58 cases had diarrhea, with the incidence of 48.33%. It may be that the definition of diarrhea was different, so the diarrhea rate was overestimated. Ferrie et al. [12] defined diarrhea as follows: continuous 2 days, the number of daily defecation ≥3 times, or the number of daily un shaping stool ≥3 times, or the number of daily defecation ≥3 times and the amount ≥300 ml/d. Diarrhea is defined by the World Health Organization as ≥ 3 times of unformed stools per day [13]. According to the 2018 British Adult Chronic Diarrhea Survey Guide, chronic diarrhea is defined as follows: unshaping stool ≥3 times a day for more than 4 weeks [14]. Diarrhea defined in this study meets the following three conditions: defecation frequency ≥3 times/d, fecal volume ≥200 g/d, fecal nature is paste or water sample (Bristol stool type 5–7). The study was a retrospective study. The treatment time of the included severe patients receiving enteral nutrition was not limited, so the observation time was long and the sample size was small, which may be an important reason for the overestimation of diarrhea rate.

Analysis of influencing factors of diarrhea during EN in ICU patients: Single factor analysis showed that there were significant differences in age, antibiotic use, ICU hospitalization time, and mechanical ventilation time between patients with diarrhea and those without diarrhea. The above indicators were further analyzed by multivariate logistic regression analysis, and the results confirmed that age ≥60 years old, the use of antibiotics, ICU hospitalization time, and mechanical ventilation time were independent risk factors for diarrhea in ICU patients during EN intervention. The dynamic balance of gastrointestinal microorganisms maintains human health. Firmicutes and Bacteroidetes in the intestine can control the amount of carbohydrates in the human body through fermentation, and the short-chain fatty acids of the fermentation products can absorb more liquids and electrolytes in the body. Once this function is destroyed, the accumulated metabolites accumulate, leading to osmotic effect and diarrhea [15]. Clinically, patients with diarrhea showed a higher number of Clostridium and a lower number of Bifidobacterium, and the imbalance of these two flora may be related to its pathogenesis. The number of bifidobacteria is a beneficial bacterium in the intestine, and the decrease in this number will reduce the inhibitory ability of the gastrointestinal tract to pathogens to some extent, such as increasing the risk of *Clostridium difficile* infection [16]. Thibault et al. [17] pointed out that antibiotics were an independent risk factor for diarrhea in patients. The use of antibiotics can provide environmental support for the reproduction and infection of *Clostridium difficile*. It can also lead to the disorder of intestinal probiotics, cause intestinal allergy, release antimicrobial toxins, increase gastric motility, and lead to nutrient absorption disorders, thereby causing diarrhea [18]. Previous studies have shown that antibiotic use is an important risk factor for nosocomial diarrhea [19, 20]. A recent study has shown that the diversity of gut microbiome is affected by antibiotic administration, and gut microbiome composition changes over time [21]. Our study found that 58% (46/73) of the same patients who used antibiotics developed diarrhea. At present, there are still controversial results on the effect of age on EN treatment intolerance [10, 22]. Our results suggest that increased age may be a risk factor for diarrhea in critically ill patients. The higher the patient's age, the lower their own immunity, reactivity and reserve capacity, and the degenerative changes in organ physiological function. The intestinal villi and microvilli of elderly patients are sparse, thick and short, and the mucosa is thin. In addition, the mitochondria of elderly patients are prone to swelling, fracture, and dissolution [23]. Compared with young people, the proportion of beneficial bacteria in fecal samples of the elderly, such as thick-walled bacteria, Clostridium, and Lactobacillus, is reduced, and the number of pathogenic bacteria such as Streptococcus and Staphylococcus is increased [24]. In addition, the elderly are at high risk for antibiotic-associated diarrhea. Antibiotic treatment based on enteral nutrition support will also increase the risk of antibiotic-associated diarrhea. There is no report on the correlation between ICU hospitalization time and diarrhea in critically ill patients treated with EN. But it is certain that the longer the ICU hospitalization time, the more complex the condition, the higher the body consumption, the longer the EN treatment of gastrointestinal dysfunction, and the higher the risk of diarrhea. The gastrointestinal motility of ICU patients is weak, and mechanical ventilation will further reduce their gastric motility function. The longer the duration of mechanical ventilation, the greater the impact on gastric motility, and the higher the incidence of diarrhea. In addition, maintaining long-term intra-abdominal pressure in patients with long-term mechanical ventilation may also be an important cause of EN treatment intolerance [22]. Heyland et al. found that patients with diarrhea did not use mechanical ventilation for a shorter period of time and had a longer hospital stay than those who were resistant to enteral nutrition [25]. In general, it is necessary to be vigilant against the occurrence of diarrhea in elderly patients who have long been in ICU during EN treatment and take timely measures. In addition, patients receiving EN treatment during mechanical ventilation should also be paid more attention, and the use of antibiotics should be reduced as much as possible during treatment. There are still many limitations in this study. Firstly, this is a single-center retrospective study, so the sample size is small and the results may be biased. Secondly, the data collected in the study were not comprehensive, and the relationship between diabetes history, enteral nutrition temperature, fasting before intervention, and diarrhea was not studied. Therefore, the risk factors may be small.

RETRACTED

## 5. Conclusion

In summary, older age, frequent use of antibiotics, long ICU stay, and mechanical ventilation time can lead to diarrhea in ICU patients receiving EN treatment. It is necessary to effectively analyze the above independent factors and implement targeted interventions to improve the incidence of diarrhea in patients.

## Figures and Tables

**Figure 1:** Flow chart for inclusion in the study.

**Figure 2:** Proportion of diarrhoea cases in patients aged ≥60 years and on antimicrobials. (a) Proportion of diarrhea in patients aged ≥60 years old. (b) Proportion of diarrhea in patients using antibiotics.

**Figure 3:** Correlation between ICU hospitalization time, mechanical ventilation time, and diarrhea risk. (a) The correlation between ICU hospitalization time and diarrhea condition. (b) The correlation between the duration of mechanical ventilation and diarrhea condition.

**Figure 4:** ROC curve for diagnosis of diarrhea.

**Table 1:** Clinical characteristic of patients.

Characteristics	Value
No. of diarrhea patients	58 (48.33)
Male sex, *n* (%)	73 (60.83)
Hypoproteinemia, *n* (%)	67 (55.83)
Use of antibiotics, *n* (%)	79 (65.83)
Mechanical ventilation, *n* (%)	95 (79.17)
BMI (kg/m^2^, mean ± SD)	21.71 ± 3.01
APACHE II score (mean ± SD)	20.31 ± 6.24
ICU hospitalization time (d, mean ± SD)	9.22 ± 2.81
Duration of mechanical ventilation (d, mean ± SD)	7.46 ± 1.95

Age, years, *n* (%)	
≥60	71 (59.17)
<60	49 (40.83)

Feeding patterns, *n* (%)	
Nasogastric tube	110 (91.67)
Nasojejunal tube	10 (8.33)

EN preparation, *n* (%)	
Integral protein	105 (87.50)
Oligopeptide	15 (12.50)

Days of EN treatment, *n* (%)	
4 days	105 (87.50)
7 days	15 (12.50)

Amount of EN (mL, mean ± SD)	
4 days	1033.49 ± 206.64
7 days	1212.47 ± 240.31

ICU admission diagnosis, *n* (%)	
Central nervous system	12 (10.00)
Respiratory system	74 (61.67)
Cardiovascular system	16 (13.33)
Postoperation	11 (9.17)
Others	7 (5.83)

Electrolyte (mmol/L, mean ± SD)	
K	4.64 ± 1.20
Na	137.15 ± 8.72
CI	97.44 ± 9.86
Ca	2.22 ± 0.59
Mg	0.74 ± 0.19

**Table 2:** Single factor analysis of diarrhea condition.

Characteristics	Diarrhea group (*n* = 58)	Nondiarrhea group (*n* = 62)	*P V*alue
Male sex, *n* (%)	38 (65.52)	35 (56.45)	0.309
BMI (kg/m^2^, mean ± SD)	21.87 ± 2.93	21.55 ± 3.09	0.569
APACHE II score (mean ± SD)	20.38 ± 6.14	20.24 ± 6.39	0.905
ICU hospitalization time (d, mean ± SD)	10.24 ± 3.03	8.26 ± 2.21	<0.001
Duration of mechanical ventilation (d, mean ± SD)	7.86 ± 1.99	7.08 ± 1.85	0.028

Age, years, *n* (%)			0.013
≥60	41 (70.69)	30 (48.39)	
<60	17 (29.31)	32 (51.61)	

Hypoproteinemia, *n* (%)			0.888
Yes	32 (55.17)	35 (56.45)	
No	26 (44.83)	27 (43.55)	

Use of antibiotics, *n* (%)			0.003
Yes	46 (79.31)	33 (53.23)	
No	12 (20.69)	29 (46.77)	

Mechanical ventilation			0.078
Yes	16 (27.59)	9 (14.52)	
No	42 (72.41)	53 (85.48)	

Feeding patterns, *n* (%)			0.582
Nasogastric tube	54 (93.10)	56 (90.32)	
Nasojejunal tube	4 (6.90)	6 (9.68)	

EN preparation, *n* (%)			0.679
Integral protein	50 (86.21)	55 (88.71)	
Oligopeptide	8 (13.79)	7 (11.29)	

Days of EN treatment, *n* (%)			0.073
4 days	54 (93.10)	51 (82.26)	
7 days	4 (6.90)	11 (17.74)	

Amount of EN (mL, mean ± SD)			
4 days	1042.29 ± 203.22	1025.26 ± 211.11	0.654
7 days	1227.50 ± 225.48	1198.40 ± 254.42	0.510

ICU admission diagnosis, *n* (%)			0.754
Central nervous system	4 (6.90)	8 (12.90)	
Respiratory system	35 (60.34)	39 (62.90)	
Cardiovascular system	9 (15.52)	7 (11.29)	
Postoperation	6 (10.34)	5 (8.06)	
Others	4 (6.90)	3 (5.17)	

Electrolyte (mmol/L, mean ± SD)			
K	4.52 ± 1.03	4.76 ± 1.33	0.272
Na	135.75 ± 6.67	138.47 ± 10.16	0.087
CI	98.54 ± 6.24	96.42 ± 12.29	0.239
Ca	2.15 ± 0.54	2.28 ± 0.63	0.220
Mg	0.73 ± 0.22	0.75 ± 0.15	0.546

RETRACTED

**Table 3:** Variable valuation.

Factors	Variables	Valuation
Age	X1	0 = <60 years, 1 = ≥60 years
Use of antibiotics	X2	0 = no, 1 = yes
ICU hospitalization time	X3	Actual values
Mechanical ventilation time	X4	Actual values

**Table 4:** Multivariate logistic regression analysis results.

Variable	*β*	Wald *χ*^2^	*P* value	OR (95% CI)
Age (1 = ≥60 years)	0.955	4.861	0.027	2.599 (1.112∼6.074)
Use of antibiotics (1 = Yes)	1.252	7.366	0.007	3.496 (1.416∼8.632)
ICU hospitalization time	0.271	10.486	0.001	1.311 (1.113∼1.544)
Mechanical ventilation time	0.241	4.442	0.035	1.273 (1.017∼1.593)

**Table 5:** ROC curve parameters.

Factors	Cutoff (d)	AUC	Youden index	Sensitivity (%)	Specificity (%)	*P* value	95%CI
ICU hospitalization time	9.5	0.710	0.361	60.3	75.8	<0.001	0.616–0.804
Mechanical ventilation time	8.5	0.632	0.253	41.4	83.9	0.013	0.531–0.732

## Data Availability

The data used to support the findings of this study are available from the corresponding author upon request.
